# Spermidine/spermine N^1^-acetyltransferase regulates cell growth and metastasis *via* AKT/β-catenin signaling pathways in hepatocellular and colorectal carcinoma cells

**DOI:** 10.18632/oncotarget.13582

**Published:** 2016-11-25

**Authors:** Cong Wang, Ping Ruan, Ying Zhao, Xiaomin Li, Jun Wang, Xiaoxiao Wu, Tong Liu, Shasha Wang, Jiuzhou Hou, Wei Li, Qian Li, Jinghua Li, Fujun Dai, Dong Fang, Chaojie Wang, Songqiang Xie

**Affiliations:** ^1^ Institute of Chemical Biology, College of Pharmacy, Henan University, Kaifeng, 475004, China; ^2^ The Key Laboratory of Natural Medicine and Immuno-Engineering, Henan University, Kaifeng, 475004, China

**Keywords:** SSAT, polyamine, metastasis, AKT, β-catenin

## Abstract

Hepatocellular carcinoma (HCC) and colorectal cancer (CRC) are among the most common cancers across the world. Therefore, identifying the potential molecular mechanisms that promote HCC and CRC progression and metastasis are urgently needed. Spermidine/spermine N^1^-acetyltransferase (SSAT) is a catabolic enzyme that acetylates the high-order polyamines spermine and spermidine, thus decreasing the cellular content of polyamines. Several publications have suggested that depletion of intracellular polyamines inhibited tumor progression and metastasis in various cancer cells. However, whether and how SSAT regulates cell growth, migration and invasion in hepatocellular and colorectal carcinoma cells remains unclear. In this study, depletion of polyamines mediated by SSAT not only attenuated the tumor cell proliferation but also dramatically inhibited cell migration and invasion in hepatocellular and colorectal carcinoma cells. Subsequent investigations revealed introduction of SSAT into HepG2, SMMC7721 hepatocellular carcinoma cells and HCT116 colorectal carcinoma cells significantly suppressed p-AKT, p-GSK3β expression as well as β-catenin nuclear translocation, while inhibition of GSK3β activity or exogenous polyamines could restore SSAT-induced decreases in the protein expression of p-AKT, p-GSK3β and β-catenin. Conversely, knockdown of SSAT in Bel7402 hepatocellular carcinoma cells and HT-29 colorectal carcinoma cells which expressed high levels of SSAT endogenously significantly promoted the expression of p-AKT, p-GSK3β as well as β-catenin nuclear translocation. Taken together, our results indicated depletion of polyamines by SSAT significantly inhibited cell proliferation, migration and invasion through AKT/GSK3β/β-catenin signaling pathway in hepatocellular carcinoma and colorectal cancer cells.

## INTRODUCTION

Hepatocellular carcinoma (HCC) and colorectal cancer (CRC) are among the most common cancers across the world [1, 2]. Particularly, nearly 25% of patients with CRC present with synchronous liver metastases at the time of initial diagnosis and 50%-75% of patients within three years after primary colonic surgery at the time of disease recurrence [3]. Despite some advances in early detection and the use of modern surgical techniques in combination with radiotherapy and chemotherapy, the prognosis of the patients with HCC and CRC still remains poor to date [4, 5]. Therefore, identifying the potential molecular mechanisms that promote HCC and CRC progression and metastasis are urgently needed.

The polyamines, including spermine, spermidine, and putrescine are ubiquitous in living organisms which are considered essential elements for cell proliferation, differentiation and growth in normal and cancer cells [6, 7]. It has been well established that an increase in intracellular polyamine concentration correlates with increased cell proliferation as well as tumorigenesis. For example, increased polyamine concentrations are often observed in the blood and urine of cancer patients, and these increased levels have been shown to correlate with poor prognosis [8–11]. Depletion of the intracellular polyamine pools using either a polyamine synthesis inhibitor or a polyamine analog invariably inhibits cell growth in breast, colon, prostate and skin cancers [12–16].

Spermidine/spermine N^1^-acetyltransferase (SSAT) is a polyamine acetyltransferase that catalyses the formation of N^1^-acetylspermine or N^1^-acetylspermidine by transferring the acetyl group from acetyl-coenzyme A to the N^1^ position of spermine or spermidine, respectively[17]. The corresponding N^1^-acetyl derivatives are either excreted outwards, or undergo further metabolism by polyamine oxidase, thus decreasing the cellular content of polyamines [17, 18]. A series of publications have suggested that SSAT play a critical role in the regulation of tumor progression and metastasis. For example, overexpression of SSAT correlates with a progressive reduction in polyamine pools as well as total arrest in cell growth in mammalian cells [19–21]. However, it is still unclear how SSAT was involved in regulating cell growth, migration and invasion in hepatocellular and colorectal carcinoma cells.

It had been reported that depletion of polyamines induced by increased SSAT expression was associated with decreased expression of AKT which plays an essential role in cancer cells growth, polarity, migration and invasion [20, 22–24]. In addition, intracellular polyamines reduction also decreases β-catenin nuclear translocation, which is accompanied by a decrease in intestinal epithelial cell migration [25]. Therefore, we used in vitro approaches to investigate whether and how AKT and β-catenin play a vital role in SSAT-mediated cell growth, migration and invasion in hepatocellular and colorectal carcinoma cells. In this study, our results suggested that depletion of polyamines by SSAT overexpression significantly decreases cell proliferation, migration and invasion through suppression of AKT/GSK3β/β-catenin signaling pathway in hepatocellular and colorectal carcinoma cells.

## RESULTS

### Intracellular concentration of polyamine is tightly regulated by SSAT

To determine the possible role of SSAT in hepatocellular and colorectal carcinoma cells, we first observed SSAT protein expression in three hepatocellular carcinoma cell lines and two colorectal carcinoma cell lines using Western blot assay. Our results showed that in HCC cell lines the protein expression of SSAT in SMMC7721, HepG2 cells was lower than in Bel7402 cells, while in colorectal carcinoma cells the protein expression of SSAT in HCT-116 cells was less than in HT-29 cells (Figure 1A). Next, we transfected the plasmid of pIRES2-SSAT or Vector into SMMC7721, HepG2 and HCT116 cells and selected stably transfected cells with G418 for at least 2 weeks. During the experiments, we selected two SSAT stably transfected cell colonies from each cell lines and examined the protein expression of SSAT. As Figure 1B shown, the protein expression of SSAT in SMMC7721, HepG2 and HCT116 cells transfected with SSAT were significantly up-regulated compared with the cells transfected with Vector. In addition, we also used two different specific siRNA to knock down SSAT expression in Bel7402 hepatocellular carcinoma cells and HT-29 colorectal carcinoma cells which expressed high levels of SSAT endogenously. After incubation with 20 nM specific siRNA for 24 h, the silencing effect was analyzed by western blot analysis, as Figure 2A shown the protein expression of SSAT was decreased significantly in cells treated with SSAT-targeted siRNA compared with the cells treated with non-sense siRNA.

**Figure 1:** SSAT over-expression down-regulated the content of polyamines in hepatocellular and colorectal carcinoma cells **A.** Western blot analysis determined the level of SSAT in three hepatocellular carcinoma cell lines (Hep G2, SMMC7721 and Bel7402) and two colorectal carcinoma cell lines (HCT 116, HT-29). **B.** Western blot analysis demonstrated that SSAT was upregulated in Hep G2, SMMC7721 and HCT 116 cells after stably transfection. Two stably transfected cell clonies were selected in each cell lines. β-actin was used as internal control. **C.** HPLC analysis showed the concentration of polyamines including spermidine and spermine were significantly down-regulated in HepG2, SMMC7721 and HCT116 cells transfected with SSAT compared with the cells transfected with Vector. While the acetylated polyamine including N^1^-acetylspermidine, N^1^-acetylspermine were profoundly increased in HepG2, SMMC7721 and HCT 116 cells transfected with SSAT compared with the cells transfected with Vector. All of the experiments were repeated three times and data was presented as means ± SEM (n=3). *p< 0.05, **p<0.01, ***p<0.001 compared to the vector group. ^#^p< 0.05, ^##^p<0.01, ^###^p<0.001 compared to the vector group, one way ANOVA.

**Figure 2:** Knockdown of SSAT up-regulated the content of polyamines in hepatocellular and colorectal carcinoma cells **A.** Western blot analysis demonstrated that SSAT was downregulated in Bel7402 and HT29 cells after treatment with two different specific SSAT siRNA. **B.** HPLC analysis showed spermidine and spermine were significantly up-regulated in Bel7402 and HT29 cells transfected with SSAT siRNA compared with the cells transfected with non-sense siRNA. While the acetylated polyamine including N^1^-acetylspermidine, N^1^-acetylspermine were profoundly decreased in Bel7402 and HT29 cells transfected with SSAT siRNA compared with the cells transfected with non-sense siRNA. All of the experiments were repeated three times and data was presented as means ± SEM (n=3). *p< 0.05, **p<0.01, ***p<0.001 compared to the vector group. ^#^p< 0.05, ^##^p<0.01, ^###^p<0.001 compared to the vector group, one way ANOVA.

As a catabolic enzyme, SSAT catalyzes acetylation of spermidine (SPD) and spermine (SPM) to generate N^1^-acetylspermidine, N^1^-acetylspermine which in turn is oxidatively degraded by acetylpolyamine oxidase (APAO) to N-acetylaminopropanal and a lower polyamine [17]. Therefore the accurate effects of SSAT on cellular polyamine metabolism were evaluated in hepatocellular and colorectal carcinoma cells. Using HPLC assay, we detected the intracellular levels of putrescine (PUT), spermidine (SPD) and spermine (SPM) in cancer cells, independently. The concentration of polyamines including spermidine and spermine were significantly down-regulated in SMMC7721, HepG2 and HCT116 cells that stably transfected with SSAT as compared with the cells transfected with Vector (Figure 1C). In addition, we also observed a decrease in the concentration of putrescine in SMMC7721, HepG2 cells (Figure 1C). Conversely, the concentrations of spermidine and spermine were significantly up-regulated in Bel7402 and HT-29 cells after knockdown of SSAT using two different siRNA (Figure 2B). Consistent with SSAT enzymatic function, acetylated polyamine including N^1^-acetylspermidine, N^1^-acetylspermine were profoundly increased in SMMC7721, HepG2 and HCT116 cells transfected with SSAT compared with the cells transfected with Vector (Figure 1C), while N^1^-acetylspermidine, N^1^-acetylspermine were decreased significantly in Bel7402 and HT-29 cells treatment with SSAT-targeted siRNA compared with the cells treated with non-sense siRNA and non-transfected cells (Figure 2B).

### SSAT inhibits cell colony formation and proliferation rate in hepatocellular and colorectal carcinoma cells

To investigate whether SSAT regulate tumor cells colony formation and proliferation, cell colony formation assay and the MTT assay were performed *in vitro*. The colony formation assay noted that overexpression of SSAT significantly inhibited the colony formation of SMMC7721, HepG2 and HCT 116 cells compared with the cells transfected with Vector (Figure 3A). Then, we investigated whether SSAT regulates cell proliferation. As Figure 3B shown when SSAT was overexpressed in SMMC7721, HepG2 and HCT116 cells, a decreased proliferation rate occurred compared with the cells transfected with Vector. Next, we wondered if loss of SSAT may promote tumor cell proliferation. Therefore, SSAT was knocked down using two different spcific SSAT-targeted siRNA and cell proliferation rate was assessed in Bel7402 and HT-29 cells which expressed high levels of SSAT endogenously. As shown in Figure 3C, a significant increased proliferation rate was observed in Bel7402 and HT-29 cells transfected with SSAT siRNA compared with control group. These results indicated that overexpression of SSAT inhibited cell colony formation and proliferation rate in hepatocellular and colorectal carcinoma cells.

**Figure 3:** SSAT was involved in cell colony formation and proliferation in hepatocellular and colorectal carcinoma cells **A.** Cell colony formation results showed enforced expression of SSAT inhibited the colony formation in HepG2, SMMC7721 and HCT 116 cells compared with cells transfected with Vector. **B, C.** MTT assay showed SSAT over-expression attenuated the cell proliferation in HepG2, SMMC7721 and HCT 116 cells, whereas knockdown of SSAT by siRNA enhanced cell proliferation in Bel7402 and HT-29 cells. Representative images were shown. All of the experiments were repeated three times and data was presented as means ± SEM (n=3). *, p< 0.05, **, p<0.01 and ***, p<0.001 compared to the control group.

### SSAT regulates cancer cells migration and invasion

In addition to investigate the anti-proliferative effects of SSAT in hepatocellular and colorectal carcinoma cells, we also asked whether SSAT regulated cancer cell migration and invasion in these cells. First, we examined the role of SSAT in tumor cell migration by using wound scratch assay. As Figure 4A shown that the cells transfected with SSAT displayed a decreased ability in wound closure compared with the cells transfected with Vector in SMMC7721, HepG2 and HCT116 cells. To further identify these observations, we examined the effects of SSAT on cell migration using the Boyden chamber transwell without Martrigel. Consistent with wound scratch assay, SMMC7721 HepG2 and HCT116 cells transfected with SSAT displayed a weaker ability of migration compared with the cells transfected with Vector (Figure 4B). Next, to determine the role of SSAT in tumor cell invasion, we performed the experiments using transwell chamber with Matrigel. As illustrated in Figure 4C, overexpression of SSAT in SMMC7721, HepG2 and HCT 116 cells significantly attenuated the cell numbers that invaded through Matrigel in comparison with the cells transfected with Vector. In contrast, knockdown of SSAT in Bel7402 and HT-29 cells enhanced cells migration and invasion compared with the cells treated with non-sense siRNA using wound scratch assay and transwell assay (Figure 5A–5C). These results indicated that SSAT play an inhibitory role in cell migration and invasion in hepatocellular and colorectal carcinoma cells.

**Figure 4:** Up-regulation of SSAT inhibited cell migration and invasion in hepatocellular and colorectal carcinoma cells **A.** Wound healing assay indicated that SSAT up-regulation promoted HepG2, SMMC7721 and HCT116 cells migration. **B, C.** Transwell chamber without (B) or with Matrigel (C) were employed to examine the migration and invasion ability of tumor cells. Cells were harvested and added in serum-free media into the top chambers. After 24 h migration or invasion, the cells on the lower surface of the filters were stained. Note that up-regulation of SSAT significantly enhanced cell migration and invasion in HepG2, SMMC7721 and HCT 116 cells. Representative images and the number of migrated or invaded cells were shown. All of the experiments were repeated at least three times and data was presented as means ± SEM. *p<0.05, **p<0.01, ***p<0.001 compared to the control group, one-way ANOVA.

**Figure 5:** Knockdown of SSAT enhanced cell migration and invasion in hepatocellular and colorectal carcinoma cells **A.** Wound healing assays revealed that knockdown of SSAT inhibited cell migration in Bel7402 and HT-29 cells. **B, C.** Knockdown of SSAT attenuated the migration and invasion in Bel7402 and HT-29 cells. Bel7402 or HT-29 cells without transfection or transfected with non-sense siRNA or SSAT specific siRNA were seeded into the transwell chamber coated without (B) or with Matrigel (C) and incubated in RPMI1640 containing 10% FBS for 24 h. Representative images were shown. All of the experiments were repeated at least three times and data was presented as means ± SEM. *p< 0.05, **p<0.01, ***p<0.001 compared to the control group, one-way ANOVA.

### AKT/β-catenin signaling pathway was vital in SSAT-regulated cell proliferation, migration and invasion

It had been reported that overexpression of SSAT induced by N^1^, N^11^-diethylnorspermine (DENSPM), a polyamine analog, inhibited the activity of AKT in glioblastoma [20]. Accumulating evidence suggested AKT was implicated in cellular processes such as cell survival, growth, migration and cell cycle progression [22, 24, 26]. Therefore, we first examined whether overexpression of SSAT was able to inhibit AKT activity in hepatocellular and colorectal carcinoma cells. As expected, introduction of SSAT into SMMC7721, HepG2 and HCT 116 cells significantly suppressed p-AKT and AKT protein expression (Figure 6A). On the other hand, knockdown of SSAT in Bel7402 and HT-29 cells dramatically promoted the protein expression of p-AKT and AKT (Figure 7A). As one of AKT downstream targets, Glycogen synthase kinase 3β (GSK3β) could be phosphorylated at Ser9 and inactivated by AKT directly, potentially leading to Wnt-independent β-catenin stabilization which is well known to play a pivotal role in tumor invasion and metastasis in various cancer cells [27–29]. Therefore, we further investigated whether AKT/GSK3β/β-catenin signaling pathway was involved in SSAT-mediated cell proliferation, migration and invasion in hepatocellular and colorectal carcinoma cells. As our results shown overexpression of SSAT in SMMC7721, HepG2 and HCT116 cells inhibited GSK3β phosphorylation at Ser9 and β-catenin expression compared with the cells transfected with Vector (Figure 6A–6B). Meanwhile, SSAT knockdown in Bel7402 and HT-29 cells induced GSK3β Ser9 phosphorylation and β-catenin expression in comparsion with the cells untreated or transfected with non-sense siRNA (Figure 7A–7B). Considering that β-catenin translocation into the nucleus where it activates downstream target genes including c-myc, cyclin-D1 and ZEB1 to promote cell proliferation, migration, invasion and metastasis [30, 31], we then detected nuclear translocation of β-catenin and one of its downstream target genes cyclin D1 expression in hepatocellular and colorectal carcinomas. As Figure 6C shown overexpression of SSAT in SMMC7721, HepG2 and HCT116 cells significantly alleviated β-catenin translocation into nucleus and cyclin D1 expression compared with the cells transfected with Vector. In contrast, β-catenin nuclear accumulation and cyclin D1 expression increased in Bel7402 and HT-29 cells transfected with two different SSAT-targeted siRNA (Figure 7C).

**Figure 6:** Up-regulation of SSAT inhibited AKT/GSK3β/β-catenin signaling pathway and Epithelial-to-Mesenchymal transition in hepatocellular and colorectal carcinoma cells **A.** Western blot analysis demonstrated that the protein expression of p-AKT, AKT and p-GSK3 was decreased in HepG2, SMMC7721 and HCT 116 cells transfected with SSAT compared with the cells without transfection or transfected with Vector. β-actin was used as an internal control. **B, C.** Western blot analysis showed the expression of β-catenin (total and nucleus protein), cyclin D1, N-cadherin, Slug and Twist1 were decreased in SMMC7721, HepG2 and HCT 116 cells transfected with SSAT compared with the cells without transfection or transfected with Vector. The epithelial marker E-cadherin was increased in HepG2, SMMC7721 and HCT 116 cells transfected with SSAT compared with the cells without transfection or transfected with Vector. Lamin B1 was used as an internal control of nucleus protein, β-actin was used as an internal control of total protein.

**Figure 7:** Silencing of SSAT induced AKT/GSK3β/β-catenin signaling pathway and Epithelial-to-Mesenchymal transition in hepatocellular and colorectal carcinoma cells **A.** Western blot analysis demonstrated that the protein expression of p-AKT, AKT and p-GSK3 was increased in Bel7402 and HT-29 cells transfected with SSAT siRNA compared with the cells transfected with non-sense siRNA. β-actin was used as an internal control. **B, C.** Western blot analysis showed the expression of β-catenin (total and nucleus protein), cyclin D1, N-cadherin, Slug and Twist1 was increased in Bel7402 and HT-29 cells transfected with SSAT siRNA compared with the cells transfected with non-sense siRNA. The expression of N-cadherin was decreased in Bel7402 and HT-29 cells transfected with SSAT siRNA. Lamin B1 was used as an internal control of nucleus protein, β-actin was used as an internal control of total protein.

According to previous reports, nuclear β-catenin binds to members of the TCF/LEF family of transcription factors to promote Epithelial-to-Mesenchymal transition (EMT) which is an essential physiological process characterized by well-defined features such as the loss of epithelial marker E-cadherin, the gain of mesenchymal cell markers N-cadherin, Snail, Slug and Twist1 [32, 33]. Therefore, we then examined the protein expression of several EMT markers in the present study. As the results shown overexpression of SSAT in SMMC7721, HepG2 and HCT116 cells significantly increased the protein expression of E-cadherin but decreased the protein expression of N-cadherin, Slug, Twist (Figure 6B–6C). While knockdown of SSAT using specific siRNA in Bel7402 and HT-29 cells abolished E-cadherin and promoted the expression of N-cadherin, Slug, Twist (Figure 7B–7C).

### GSK3β is an important mediator in AKT/β-catenin signaling pathway

As mentioned above, overexpression of SSAT in SMMC7721, HepG2 and HCT116 cells alleviated the protein expression of p-AKT, p-GSK3β and β-catenin. To further characterize GSK3β is an important mediator in AKT/β-catenin signaling pathway, we used Lithium chloride (LiCl) which is known to activate canonical Wnt signaling by inhibiting glycogen synthetase kinase3β to monitor the activity of β-catenin. Meanwhile, we also observed GSK3β kinase activity by measuring the phosphorylation levels of GSK3β at Ser9 which is an indicator of GSK3β inactivation. Our results showed that after treatment with 5 mM LiCl for 48 h, the expression of phosphorylated GSK3β was increased in SMMC7721, HepG2 and HCT116 cells transfected with SSAT (Figure 8A). Additionally, a significant increase of β-catenin total protein appeared compared with the control group without LiCl treatment (Figure 8A). These results indicated that GSK3β is a negative mediator in AKT/β-catenin signaling pathway. In order to investigate whether inhibition of GSK3β activity could restore SSAT-induced cell growth and invasion progress in hepatocellular and colorectal carcinoma cells, we then performed the MTT cell viability assay and Boyden chamber transwell assay in the absence or presence of LiCl in SMMC7721, HepG2 and HCT116 cells transfected with SSAT. The results revealed that LiCl could reverse SSAT-induced cell growth inhibition and decreases in the cell number invaded through Matrigel (Figure 8B–8C).

**Figure 8:** The GSK3β inhibitor LiCl reversed SSAT-induced inhibition of AKT/β-catenin signaling pathway as well as cell proliferation, migration and invasion in hepatocellular and colorectal carcinoma cells **A.** Western blot analysis showed GSK 3β inhibitor LiCl markedly reversed SSAT-induced p-GSK3β and β-catenin down-regulation in SMMC7721, HepG2 and HCT116 cells transfected with SSAT. β-actin served as an internal control. **B.** MTT assay showed LiCl attenuated SSAT-induced inhibition of cell proliferation in SMMC7721 (a), HepG2 (b) and HCT 116 cells (c). *p< 0.05, **p<0.01, ***p<0.001 compared to the control group, one-way ANOVA. **C.** Transwell assay with Matrigel demonstrated LiCl restored SSAT-induced inhibition of cell invasion in SMMC7721, HepG2 and HCT 116 cells. *p< 0.05, **p<0.01, ***p<0.001 compared to the control group, one-way ANOVA.

### Inhibition of cell growth and invasion in HepG2, SMMC7721 and HCT 116 cells transfected with SSAT is due to depletion of polyamines

As our results shown, SSAT overexpression or knockdown could alter cell growth rate, migration and invasion in hepatocellular and colorectal carcinoma cells. To distinguish the effects of signaling pathways from the effects of altered polyamine levels on cell behaviors, we first treated SSAT-transfected cells with polyamines for 3 days and detected the protein expression of p-AKT, AKT, p-GSK3β and β-catenin. As shown in Figure 9A, exogenous polyamines (PUT 0.08 μM, SPD 0.5 μM, SPM 1.0 μM) restored SSAT-induced decreases in the expression of p-AKT, AKT, p-GSK3β and β-catenin in SMMC7721, HepG2 and HCT 116 cells transfected with SSAT. In order to identify polyamine depletion induced by SSAT was involved in regulating cell growth, migration and invasion, we performed the MTT cell viability assay in the absence or presence of exogenous polyamines in SMMC7721, HepG2 and HCT 116 cells transfected with SSAT, the results revealed that exogenous polyamines could reverse SSAT-induced cell growth inhibition 9B. Besides, we also examined cells invasion using the Boyden chamber transwell assay. As illustrated in Figure 9C, polyamines (PUT, SPD, SPM) supplementation significantly reversed SSAT-induced decreases in the cell number invaded through Matrigel. Taken together, these findings support the conclusion that depletion of polyamines by SSAT significantly decreases cell proliferation, migration and invasion through the suppression of AKT/GSK3β/β-catenin signaling pathway in hepatocellular and colorectal carcinoma cells.

**Figure 9:** The exogenous polyamines (PUT, SPD, SPM) reversed SSAT-induced inhibition AKT/β-catenin signaling pathway as well as cell proliferation and invasion in hepatocellular and colorectal carcinoma cells **A.** Western blot analysis showed exogenous polyamines reversed SSAT-induced p-AKT, AKT, p-GSK3β and β-catenin down-regulation in HepG2, SMMC7721 and HCT116 cells transfected with SSAT. β-actin served as an internal control. **B.** MTT assay showed exogenous polyamines attenuated SSAT-induced inhibition of cell proliferation in SMMC7721 (a), HepG2 (b) and HCT 116 cells (c). *p< 0.05, **p<0.01, ***p<0.001 compared to the control group, one-way ANOVA. **C.** Transwell assay with Matrigel demonstrated exogenous polyamines restored SSAT-induced inhibition of cell invasion in SMMC7721, HepG2 and HCT 116 cells. *p< 0.05, **p<0.01, ***p<0.001 compared to the control group, one-way ANOVA.

## DISCUSSION

Polyamines are essential for normal cell growth and differenation, and aberrant polyamine metabolism is known to play an important role in the development of tumors [34, 35]. SSAT is the principal catabolic enzyme responsible for the regulation of intracellular polyamine contents in mammalian cells. Recent studies have indicated that chemotherapeutic agents, such as cisplatin, paclitaxel, doxorubicin, 5-FU and oxaliplatin may induce SSAT expression and decrease total polyamines content in cells [36–39]. In this study, we found the concentration of spermidine and spermine was significantly decreased in SMMC7721, HepG2 and HCT116 cells transfected with SSAT. Accordingly, knockdown of SSAT in Bel7402 and HT-29 cells produced an upregulation in spermidine and spermine. This is consistent with previous findings that overexpression of SSAT in several cell lines induced the depletion of spermidine and spermine [6, 40]. In addition, we also found a decrease of putrescine in HepG2, SMMC7721 cells transfected with SSAT. In contrast, several previous studies suggested SSAT overexpression often results in an increase of putrescine since it's the product of polyamine catabolism [17, 41]. It is noteworthy that putrescine can be converted to spermidine by S-adenosylmethionine decarboxylase (SAMDC) in polyamine-depleted cells, yielding N^1^-acetyl derivatives by SSAT which are either excreted outwards or undergo further metabolism by polyamine oxidase [17, 42]. Therefore, we speculated SSAT overexpression in a short time led to an increase of putrescine but a decrease in a long time owing to polyamines depletion. Consistent with our assumption, Morada M et al found putrescine increased by 2.5-fold after 15 h of SSAT overexpression and then decreased after 24 h in intestinal adenocarcinoma HCT-8 cells [43].

High polyamine levels have been detected in most types of cancers. For example, in colorectal cancer, the polyamine contents are increased 3- to 4-fold over those found in the equivalent normal tissue. Depletion of the intracellular polyamine pools invariably inhibits cell growth [6, 44]. Here, our findings showed depletion of polyamines induced by SSAT overexpression resulted in decreased cell proliferation in SMMC7721, HepG2 and HCT116 cells which is consisitent with previous reports that SSAT induction plays a key role in cells growth inhibition in glioblastoma cells, Caco-2 colon cancer cells, A2780 human ovarian carcinoma cells [45–47]. Although there were some studies demonstrated that the depletion of polyamines leads to growth inhibition in mammalian cells through various pathways such as a total arrest in protein translation, mitochondria-mediated apoptosis or cell cycle arrest [6, 40, 48]. However, it is still debated whether the arrest in polyamine-depleted cells occurs in G1, S or G2 or all of them.

In addition, patients with increased polyamine levels either in the blood or urine are reported to have more advanced disease and worse prognosis compared to those with low levels, regardless of the type of malignancy [9, 10]. Depletion of polyamines by treatment with DFMO, a drug that blocks the enzyme ornithine decarboxylase responsible for conversion of ornithine to putrescine, has been shown to globally inhibit cell migration, while supplementation with polyamine reverses the DFMO-induced decrease in invasive qualities [49–51]. Therefore, the rapid and extensive depletion of polyamine by SSAT transduction has permitted us to address the role of polyamines in cells migration and invasion. Using wound healing and transwell assays, we provided evidence that depletion of polyamine induced by SSAT overexpression inhibited cell migration and invasion in hepatocellular and colorectal carcinoma cells, whereas reduction of SSAT by siRNA attenuated it.

The development of HCC and CRC has been related to various altered signaling pathways, including the Wnt/β-catenin signaling pathway [52, 53]. β-catenin functions as a key transcriptional factor regulating the expression of pro-proliferation/metastasis proteinsvia aberrant expression and nuclear translocation [31, 54]. In the absence of Wnt, cytoplasmic β-catenin is phosphorylated on several serine and threonine residues by a destruction complex containing GSK3β, casein kinase1 (CK1), axin and adenomatous polyposis coli (APC), which leads to ubiquitin-proteasome-mediated degradation of β-catenin [27, 55]. Lithium chloride (LiCl) is known to activate canonical Wnt signaling by inhibiting GSK3β and consequently stabilizing free cytosolic β-catenin [56, 57]. Coincidently, in our study we found that depletion of polyamine induced by SSAT over-expression decreased p-GSK3β expression and inhibited β-catenin nuclear translocation in hepatocellular and colorectal carcinoma cells. In support of our findings, a study by Guo X et al suggested polyamine depletion by DFMO decreased the levels of total β-catenin protein leading to decreased cell migration in intestinal epithelial cells [25]. Activated AKT can block the kinase activity of GSK3β by phosphorylating GSK3β at Serine 9 leading to β-catenin nuclear accumulation. In glioblastoma, overexpression of SSAT could down-regulate AKT expression, thus resulting in cell detachment and apoptosis. In the current study, we also observed a decreased protein expression of p-AKT and AKT and a reduced cell proliferation, migration and invasion in HepG2, SMMC7721 and HCT 116 cells transfected with SSAT. In summary, these results indicated that the AKT, GSK3β and β-catenin worked together as AKT/GSK3β/β-catenin pathway regulating cell proliferation, migration and invasion in HCC and CRC. Conflicting with our results, several published papers indicated that polyamine depletion by DFMO induced AKT/GSK3β pathway in neuroblastoma and IEC-6 cells [49, 58]. Further studies confirmed that depletion of polyamines by DFMO induces two opposing pathways in these cells: one promoting cell survival by activating Akt/PKB and one inducing p27^Kip1^/retinoblastoma-coupled G1 cell cycle arrest via a mechanism that regulates the phosphorylation and stabilization of p27^Kip1^ [58, 59]. Obviously, AKT also plays a positive role in promoting cell survival in these cancer cells which is consistent with our results. Therefore, we speculated that the conflicting results may be due to the different strategies of polyamine depletion. This may explain the moderate efficacy of DFMO monotherapy in clinical trials for cancer treatment.

Chen et al have reported that overexpression of SSAT increases integrin α9β1-mediated migration, and siRNA knockdown of SSAT inhibited α9β1-dependent migration without affecting cell adhesion or migration mediated by other integrins [60]. deHart et al. further demonstrate that integrin mediates dynamic localized regulation of polyamine levels by SSAT, resulting in block of inward rectifier potassium channels, an increase in membrane potassium permeability, and stimulation of cell migration [61]. Contrast to these results, Rao JN et al found polyamine depletion inhibits Kv channel expression which downregulates cytosolic free Ca^2+^concentration and decreases cell migration [62]. In the present study, we did observe that overexpression of SSAT in hepatocellular and colorectal carcinoma cells could inhibit, not promote cells migration and invasion. Based on our results, we speculated that SSAT-mediated cell migration by binding to the integrin alpha9 subunit cytoplasmic domain does not play a critical role in these cancer cells.

In the present study, we used several cell lines to investigate the role of SSAT. Although each cell lines contain different levels of polyamines, the effect of SSAT was similar degree in all cell lines. This may because the activity of SSAT was saturated as a polyamine acetyltransferase, leading to the effect of SSAT reaching its best degree.

In conclusion, we uncover the function and mechanisms of SSAT in regulating cancer cells survival, migration and invasion in hepatocellular and colorectal carcinoma cells. The depletion of polyamines by SSAT overexpressing significantly decreases cell proliferation, migration and invasive capacity of cells through the suppression of AKT/GSK 3β/β-catenin pathway, suggesting its possible application as a molecular target for therapy.

## MATERIALS AND METHODS

### Materials

3-(4, 5-dimethylthiazol)-2, 5-diphenyltetrazolium bromide (MTT), G418, putrescine, spermine, spermidine and LiCl were purchased from Sigma (St. Louis, MO, USA). RPMI 1640 and fetal bovine serum (FBS) were purchased from Gibco (Grand Island, NY, USA). The sources of primary antibodies used for Western blot: AKT (cat. sc-5298), p-AKT1/2/3(Ser 473) (cat. sc-7985-R), cyclin D1 (cat. sc-753), SSAT (cat. sc-67159), E-cadherin (cat. sc-31021), N-cadherin (cat. sc-7939), β-catenin (cat. sc-7199), β-Actin (cat. sc-47778) as well as the corresponding horseradish peroxidase-conjugated second antibodies were all purchased from Santa Cruz Biotechnologies (Santa Cruz, CA, USA). Phospho-GSK-3β (Ser9) (#9323) was purchased from Cell Signaling Technology. SLUG (cat. ab50887), Twist (ab27568), Lamin B1 (ab194109) were from Abcam (Cambridge, England), RIPA buffer, BCA assay kit, ECL plus reagents were purchased from Beyotime (China). All other chemicals used in this study were commercial products of reagent grade.

### Cell culture

The cells lines, derivative from human HCC (HepG2, SMMC7721, and Bel7402) and colorectal carcinoma cells (HCT116 and HT-29), were purchased from the cells bank of the Chinese Academy of Science (Shanghai, China). These cells were cultured in RPMI1640 medium supplementing with 10% FBS, 100 units/mL penicillin and 100 μg/mL streptomycin, in a humidified incubator containing 5% CO_2_ at 37°C.

### Plasmid transfection

Constructed plasmid, siRNA and negative control siRNA were prepared for transfection. For SSAT transfection, HepG2, SMMC7721 and HCT116 cells were seeded in 24-well plates at 5×10^4^ per well and cultured at 37°C in a humidified atmosphere with 5% CO_2_. The next day, when the cells were approximately 60% confluent, they were transfected with a mixture of 2 μl TurboFect™ in vitro Transfection Reagent and 1μg plasmids according to the manufacturer's instructions. After 36 h, these transfected cells with pIRES2-EGFP-SSAT or pIRES2-EGFP vector were selected through 0.4 mg/mL G418 for least 2 weeks. And then, the limiting dilution analysis was used to select the stable plasmid-transfected clones in 96-well plates. The clones derived from HepG2, SMMC-7721 and HCT 116 cells stably transfected with pIRES2-EGFP-SSAT or pIRES2-EGFP vector were classified as SSAT and Vector respectively. In this study, we selected two stably clones derived from HepG2, SMMC-7721 and HCT 116 cells transfected with pIRES2-EGFP-SSAT to perform the subsequent experiments.

For small interference RNA transfection, SSAT was disrupted by small interfering RNA, siSSAT. siSSAT oligonucleotides and corresponding scrambled oligonucleotides were purchased from Sigma (St. Louis, MO, USA). Their sequences were as follows: siRNA, sense strand 5′-GCA GCA GCA UGC ACU UCU UTT-3′, antisense strand 5′-AAG AAG UGC AUG CUG CUG CTT-3′; A scrambled sequence (served as a negative control), sense strand 5′-UUC UCC GAA CGU GUC ACG UTT-3′, antisense strand 5′-ACG UGA CAC GUU CGG AGA ATT-3′. When Bel7402 and HT-29 cells were approximately 60% confluent in a 6-well plate, transiently transfected with siSSAT oligonucleotides or scrambled oligonucleotides with 2 μl TurboFect™ in vitro Transfection Reagent. The cells transfected with siSSAT oligonucleotides or scrambled oligonucleotides transiently were named as Bel7402-siSSAT, HT-29-siSSAT, Bel7402-siControl and HT-29-siControl, respectively. After incubated for indicated time points, the transiently transfected cells were harvested for western blotting or other experiments.

### Colony formation assay

To determine the effects of SSAT overexpression on colony formation of HepG2, SMMC7721 and HCT116 cells, overexpressed SSAT-carrying and control cells were seeded in 6-well plate and incubated in RPMI1640 containing 10% FBS at a density of 400 cells per well. Cell medium was changed every 3 days for 15 days until visible colonies formed. The cell colonies (>50 cells/colony) were counted by staining with 0.1% crystal violet for 20 min. All experiments were repeated in triplicate and representative photos of the colonies were captured.

### Cell proliferation assays

The MTT assay was used to detect the proliferation rate of tumor cells. To explore the effects of SSAT on tumor cells proliferation, 2×10^2^ SSAT over-expressing or control HepG2, SMMC7721 and HCT116 cells were seeded into 96-well plates. At indicated time points, 50 μl MTT solution (1 mg/ml) was added to each well for 4 hours incubation at 37°C. After supernatants were removed from the wells, 100 μl DMSO was added to solubilize the crystal products at room temperature for 10 min. The absorbance (OD) was measured at a wavelength of 570 nm with a microplate reader (Bio-Rad). The experiments repeat at least three times. For small interference RNA transfection, Bel7402 and HT-29 cells were seeded into 96-well plates at a density of 2×10^2^ cells per well. After adherence, the cells were transfected with siSSAT oligonucleotides or scrambled oligonucleotides, respectively. Then the transiently transfected cells were used to detect the proliferation rate by MTT assay at indicated time points. To examine whether exogenous polyamines or GSK3 inhibitor LiCl could reverse SSAT-induced cell growth inhibition, we used polyamines (0.08 μM putrescine, 0.5 μM SPD, 1.0 μM SPM) or 5 mM LiCl to incubate HepG2, SMMC7721 and HCT116 cells stably transfected with SSAT for 3 days, then the cell viability was assessed by MTT assay. During incubation with polyamines, 1 mM aminoguanidine was routinely included in the media as an inhibitor of bovine serum amino oxidase to prevent oxidation of extracellular polyamines to toxic products.

### Migration and invasion assays

The migration and invasion assays were performed using a 24-well transwell chamber (8 μm poresize, polycarbonate membrane) (Corning, NY, USA) with or without Matrigel, respectively. For migration assay, 4×10^4^ cells suspended in 200 μL serum-free medium was added to the upper compartment of the transwell chamber, whereas 600 μl complete medium was placed in the lower chamber. After incubation at 37°C for 24 h, the non-migrating cells were removed with cotton swabs, which were scraped off the top of the transwell. On the lower surface of transwell chamber, the migrating cells were stained with 0.1% crystal violet after fixation and methanol. For invasion assay, the transwell was coated with Matrigel to form a matrix barrier and tumor cells were seeded only with 3×10^4^ in upper compartment. Apart from this, the other operation is same with migration assays. The number of invading or migrating cells was determined by counting four high-power fields (×100) randomly on each membrane and counted by two independent observers.

### Wound healing

Wound healing experiment was used to detect the migration ability. The cells were plated into 24-well plates and grown to create a confluent monolayer after 24 h. The cells were scratched in a straight line using a 10 μL micropipette tip (time 0) and washed with PBS and then cultured in serum-free medium. The wound of cells was visualized at 0 h, 24 h, which was observed under a phase-contrast inverted microscope.

### Polyamine determination by HPLC

The amount of natural polyamines (spermine, spermidine, putrescine) was analyzed by high performance chromatography (HPLC) in both hepatocellular and colorectal carcinoma transfected with SSAT or siSSAT. Briefly, the cells were harvested in 200 μL of PBS, and 200 μL of hexanediamine (1.624 μg/ml) was added as an internal standard. After adding 200 μL of dansyl chloride (5 mg/ml), the mixtures were incubated at 50°C for 30 min, and then the reaction was terminated by the addition of 1 mL of ethyl acetate. The supernatant containing the polyamines was functionalized with dansyl chloride and purified with an organic filtration. 20 μL of the sample was then injected onto a XDB-C18 column (4.6 ×250 mm, Agilent Technologies), which was achieved excitation at 340 nm and measured emission at 515 nm by fluorescence detector. The solvent system was consisted with methanol and water, running at 65% (v/v) to 100% (v/v) methanol with in 25 min at a flow rate of 1 mL/min. The polyamine content of cells treatment with exogenous polyamines (putrescine 0.08 μM, spermidine 0.5 μM, spermine 1.0 μM) were aslo measured in the same way.

### Western blot analysis

Western blot analysis was performed as our described previously [52]. After being washed with ice-cold phosphate buffered saline (PBS), cell pellets were lysed with RIPA buffer (Beyotime, Jiangsu, China) added along with protease inhibitor and phosphoesterase inhibitor (Roche, Basel, Switzerland). To extract nuclear proteins, the isolated nuclei were resuspended in NETN buffer (150 mM NaCl, 1 mM EDTA, 20 mM Tris-HCl (pH 8.0), 0.5% Nonidet P-40, 1 mM Na_3_VO_4_, 10 mM NaF, 1 mM phenylmethanesulfonyl fluoride and 2 μg/ml aprotinin), and the mixture was sonicated briefly to aid nuclear lysis. Nuclear lysates were collected after centrifugation at 16100 *g* for 20 min at 4°C. BCA assay kit was used to determine the concentration of protein. The total cells lysates were separated by 12% SDS-PAGE, and then transferred onto PVDF membranes. Membranes were blocked by 5% dried skimmed milk for 1 h, and then incubated with corresponding primary antibodies overnight at 4°C. After 3 washes with Tris-buffered saline with Tween (TBST), the membranes were incubated with horse-radish peroxidase (HRP)-conjugated rabbit or mouse secondary antibodies for 2 hour at room temperature. Triple-washed with TBST, bands were visualized using enhanced chemiluminescence (ECL) reagents.

### Statistical analysis

The SPSS 16.0 software (SPSS, Chicago, IL) was used for statistical analysis. Data were represented by the mean ± SME from at least three independent experiments. A two-tailed unpaired t-test was used for the comparison of the mean values between two groups. One-way analysis of variance (ANOVA) followed by Dunnett's multiple comparison test or two-way ANOVA followed by Bonferroni post-hoc test was used for multiple comparison. Differences with P<0.05 were considered statistically significant.
